# Molecular predictors of brain metastasis-related microRNAs in lung adenocarcinoma

**DOI:** 10.1371/journal.pgen.1007888

**Published:** 2019-02-01

**Authors:** Guogui Sun, Xiao Ding, Nan Bi, Zhiwu Wang, Lihong Wu, Wei Zhou, Zitong Zhao, Jingbo Wang, Weimin Zhang, Jing Fan, WenJue Zhang, Xin Dong, Ning Lv, Yongmei Song, Qimin Zhan, LuHua Wang

**Affiliations:** 1 Department of Radiation Oncology, National Cancer Center/Cancer Hospital, Chinese Academy of Medical Sciences and Peking Union Medical College, Beijing, China; 2 State Key Laboratory of Molecular Oncology, National Cancer Center/Cancer Hospital, Chinese Academy of Medical Sciences and Peking Union Medical College, Beijing, China; 3 Department of Radiation Oncology, North China University of Science and Technology Affiliated People's Hospital, Hebei, China; 4 Department of Radiation Oncology, Shandong Provincial Hospital, Shandong, China; 5 Department of Pathology, National Cancer Center/Cancer Hospital, Chinese Academy of Medical Sciences and Peking Union Medical College, Beijing, China; 6 Laboratory of Molecular Oncology, Peking University Cancer Hospital and Institute, Beijing, China; DFCI, UNITED STATES

## Abstract

Brain metastasis (BM) is a major complication of lung adenocarcinoma (LAD). An investigation of the pathogenic mechanisms of BM, as well as the identification of appropriate molecular markers, is necessary. The aim of this study was to determine the expression patterns of microRNAs (miRNAs) in LAD with BM, and to investigate the biological role of these miRNAs during tumorigenesis. miRNA array profiles were used to identify BM-associated miRNAs. These miRNAs were independently validated in 155 LAD patients. Several *in vivo* and *in vitro* assays were performed to verify the effects of miRNAs on BM. We identified six miRNAs differentially expressed in patients with BM as compared to patients with BM. Of these, miR-4270 and miR-423-3p were further investigated. miR-4270 and miR-423-3p directly targeted *MMP19* and *P21*, respectively, to influence cell viability, migration, and colony formation *in vitro*. miR-4270 downregulation and miR-423-3p upregulation was associated with an increased risk of BM in LAD patients. Thus, our results suggested that miR-4270 and miR-423-3p might play an important role in BM pathogenesis in LAD patients, and that these miRNAs might be useful prognostic and clinical treatment targets.

## Author summary

Brain metastasis (BM) is a major complication of lung carcinoma. Here, we aimed to identify the key miRNAs involved in BM lung cancer. We first profiled miRNA expression in 32 tissues from NSCLC patients with BM and 55 tissues from NSCLC patients without BM. We independently validated our results in 68 additional tissues from NSCLC patients. Based on our results, we identified a panel of miRNAs that distinguish BM lung adenocarcinomas from non-BM We report here for the first time that either miR-4270 downregulation or miR-423-3p upregulation significantly increased cell proliferation, colony formation, and migration *in vitro*. miR-4270 and miR-423-3p increased the risk of BM in mouse models by targeting *MMP19* and *P21*, respectively. Our results suggested that miR-4270 and miR-423-3p might be useful markers of BM in lung adenocarcinoma.

## Introduction

MicroRNAs (miRNAs) are small, (18–23 nt), single-stranded noncoding RNAs [1]. miRNAs play critical roles in almost all important cellular processes, including tumorigenesis [2]. Compared to long non-coding RNAs (lncRNAs; >200 nt), miRNAs are more stable *in vivo* [1–2]. As miRNAs are widely distributed in various bodily fluids, such as spit and serum, miRNA-based tumor detection techniques may have great clinical value.

Mature miRNAs combine with the 3'-UTR sequences of target genes, forming RNA-induced silence compounds; these compounds regulate gene transcription or degrade cytoplasmic mRNAs, thereby affecting protein synthesis [1–3]. Several differentially expressed miRNAs in malignant human tumors have been identified [4−6]. In general, a single miRNA can target and silence a series of target genes, granting miRNAs extensive control of various cellar processes, including proliferation, apoptosis, and tumor metastasis [7−9]. Emerging evidence indicates that miRNAs may play an important role in cancer pathogenesis [8.^9^]. Besides functioning as signal molecules in tumor tissues, exome-encoded miRNAs are also secreted in bodily fluids [10,11]. Due to the stability of miRNAs *in vivo*, miRNAs are promising candidate biomarkers for human cancers [12].

Lung cancer is one of the most aggressive malignant cancers worldwide [13]. Non-small cell lung cancer (NSCLC), the main pathological subtype of lung cancer, includes two major histologic subtypes: lung adenocarcinoma (LAD) and squamous cell carcinoma [14,15]. Despite advancements in clinical management, the overall survival of NSCLC patients remains poor, with a five-year survival rate of less than 15% [14,15]. Metastasis is the main cause of NSCLC-associated death. In addition to the lungs, NSCLC tends to metastasize in the brain, bones, and liver [16]. Brain metastasis (BM) is a frequent complication of LAD; the incidence of locally-advanced LAD with BM is as high as 30–50% [15–17]. BM is often associated with severe neurologic and cognitive difficulties, as well as disappointing survival rates [18]. Radiotherapy is the standard treatment for NSCLC-associated BM, but long-term survival remains low, with a median survival time of about 2.4–4.8 months [17,18]. Thus, it is critically important to improve patient stratification. Although the patient stratification process is greatly is greatly simplified by molecular markers, the identification of new molecular markers remains difficult. Therefore, to improve NSCLC management, it is important to identify biomarkers that enable the accurate detection of early alterations in the molecular characteristics of BM-associated tumors. Several miRNAs useful for NSCLC tumor classification, metastasis prediction, and patient prognosis have already been described [19−21]. However, it is still important and useful to identify reliable predictive miRNA markers for BM NSCLC [22].

BM occurs significantly more frequently in stage IIIA and IIIB (N2) LAD patients than in squamous patients [23,24]. Indeed, certain tumor alterations, linked to BM risk by pertinent biomarkers, could be integrated into clinical decisions as prognostic indicators, facilitating the development of personalized treatments and follow-up plans. Therefore, we focused on the regulatory roles of miRNAs in the cellular activities that impacted LAD metastasis. We also explored the use of miRNAs as biomarkers and in therapy.

## Results

### miRNA expression profiles associated with BM LAD

To identify the miRNAs associated with BM LAD, we compared miRNA expression profiles in 32 LAD patients with BM to those of 55 patients without BM (NBM) (**Table 1**). These 86 patients were considered the "discovery group." Fluorescent signals were normalized using the median center gene tool in Cluster 3.0, and evaluated using the significance analysis of microarrays (SAM) method, with a false discovery rate (FDR) threshold of 0, a fold-change of ≥2 or ≤0.5, and a *P*-value <0.05. We identified six miRNAs that were differentially expressed in the BM LAD tissues as compared to the NBM tissues (**Fig 1A, S1 Data**). Five of these miRNAs (miR-214, miR-423-5p, miR-210, miR-193a-5p, and miR-423-3p) were significantly upregulated in the BM group, while one miRNA (miR-4270) was downregulated. We validated these results in 68 BM LAD samples using quantitative real-time polymerase chain reaction (qRT-PCR). These 60 samples were considered the "validation group." The qRT-PCR results for the validation group were consistent with the analysis of the discovery group: the same six miRNAs were identified as differentially expressed (**Fig 1B; Table 1**). These results suggested that only six miRNA markers might be necessary to effectively identify BM LAD in Chinese patients.

**Fig 1:** miRNA expression profile clustering. (A) Unsupervised clustering of the miRNA expression profiles from the discovery group: 32 lung adenocarcinoma cases that developed brain metastasis (BM) and 55 BM-free cases. (B) Quantitative RT-PCR results for miR-4270, miR-214, miR-423P-5p, miR-210, miR-193-5p, and miR-423-3p in 87 samples from the discovery group. BM indicates patients with BM, and NBM indicated patients without BM. (C) Kaplan-Meier analysis of the BM-free survival of 155 patients from both the discovery and the validation groups. Patients were divided into two groups based on miRNA expression in the primary tumor. (D) Receiver operating characteristic (ROC) curve analysis of the six miRNAs that may predict BM in LAD patients.

**Table 1:** Clinical characteristics of LAD patients with and without brain metastasis.

Characteristics	Discovery group			Validation group			Full group		
	BM (n = 32)	NBM (n = 55)	*P*	BM (n = 30)	NBM (n = 38)	*P*	BM (n = 62)	NBM (n = 93)	*P*
Gender									
Male	17 (53.1%)	33 (60%)	0.532	17 (56.7%)	25 (65.8%)	0.442	34 (54.8%)	58 (62.4%)	0.350
Female	15 (46.9%)	22 (40%)		13 (43.3%)	13 (34.2%)		28 (45.2%)	35 (37.6%)	
Age									
≤ 60	20 (62.5%)	27 (49.1%)	0.226	13 (43.3%)	16 (42.1%)	0.919	33 (53.2%)	43 (46.2%)	0.394
> 60	12 (37.5%)	28 (50.9%)		17 (56.7%)	22 (57.9%)		29 (46.8%)	50 (53.7%)	
Tumor stage									
T1+ T2	27 (84.4%)	47 (85.5%)	0.892	28 (93.3%)	34 (89.5%)	0.577	55 (88.7%)	81 (87.1%)	0.764
T3	5 (15.6%)	8 (14.5%)		2 (6.7%)	4 (9.5%)		7 (11.3%)	12 (12.9%)	
Histologic grade									
Well/moderate	22 (68.8%)	34 (61.8%)	0.515	9 (30.0%)	13 (34.2%)	0.712	31 (50.0%)	46 (49.5%)	0.948
Poor/NS	10 (31.2%)	21 (38.2%)		21 (70.0%)	25 (65.8%)		31 (50.0%)	47 (50.5%)	
Lymph node ratio									
≤1/3	10 (31.2%)	26 (47.3%)	0.143	20 (66.7%)	23 (60.5%)	0.602	30 (48.4%)	49 (52.7%)	0.600
>1/3	22 (68.8%	29 (52.7%)		10 (33.3%)	15 (39.5%)		32 (51.6%)	44 (47.3%)	

BM, brain metastasis; NBM, no brain metastasis; NS, not stated.

For subsequent analyses, all samples were split into high- and low-expression groups based on the median fluorescence signal values or the qRT-PCR results for the six differentially expressed miRNAs. Univariate cox regression analyses of the discovery dataset, the validation dataset, and both datasets combined indicated that the upregulation of miR-214, miR-423-5p, miR-210, miR-193a-5p, and miR-423-3p, as well as the downregulation of miR-4270, were associated with an increased risk of BM in LAD (**Fig 1C; S1A and S1B Fig; S1 Table**). The area under the curve (AUC) values, which reflected the predictive accuracy of the six differentially expressed miRNAs, were 0.926, 0.870, and 0.902 for the discovery, validation, and combined groups, respectively (**Fig 1D**). Thus, these miRNAs accurately predicted BM in LAD patients. The sensitivity, specificity, and false discovery rate of the six micro-RNAs combined were better than those of the upregulated miRNAs alone or the downregulated miRNA alone when predicting BM with a multivariate cox regression analysis (**S2–S4 Tables**). As little is known about the roles of miR-4270 and miR-423-3p in tumor invasion and, these miRNAs were selected for further investigation [25].

### miR-4270 and miR-423-3p expression in LAD patients with BM

To investigate whether miR-4270 and miR-423-3p were suitable biomarkers of BM in LAD patients, we first analyzed miR-4270 and miR-423-3p expression levels in LAD samples. miR-4270 expression levels in NBM LAD patients were significantly higher those of BM LAD patients in all three groups (the discovery group, the validation group, and the combined group; **Table 2**). miR-4270 expression levels were not correlated with age, gender, T stage, histologic grade, or lymph node ratio (**Table 2**). Across all parameters, multivariate Cox proportional hazard regression analyses suggested that miR-4270 upregulation led to significantly positive prognostic factors, and was independent of BM in all three groups (**Table 3**). However, miR-423-3p upregulation was significantly correlated with the number of brain metastases (**Table 4**). miR-423-3p expression levels were also not correlated with age, gender, T stage, histologic grade, or lymph node ratio (**Table 4**). Multivariate cox proportional hazard regression analysis suggested that miR-423-3p upregulation was linked to poor survival in BM LAD patients, and was an independent prognostic factor for overall survival (OS) of LAD patients (**Table 5**).

**Table 2:** Correlation between miR-4270 expression and the clinicopathological features of LAD patients with and without BM.

Characteristics	miR-4270 expression levels of discovery group			miR-4270 expression levels of validation group			miR-4270 expression levels of full group		
	Low (n = 44)	High (n = 43)	*P*	Low (n = 34)	High (n = 34)	*P*	Low (n = 78)	High (n = 77)	*P*
Gender									
Male	26 (59.1%)	24 (60.5%)	0.757	21(50.0%)	21 (50.0%)	1.000	47 (60.3%)	45 (58.4%)	0.818
Female	18 (40.9%)	19 (39.5%)		13 (50.0%)	13 (50.0%)		31 (39.7%)	32 (41.6%)	
Age									
≤ 60	25 (56.8%)	22 (51.2%)	0.597	15 (44.1%)	14 (41.2%)	0.806	40 (51.3%)	36 (46.8%)	0.573
> 60	19 (43.2%)	21 (48.8%)		19 (55.9%)	20 (58.8%)		38 (48.7%)	41 (53.2%)	
Tumor stage									
T1+ T2	36 (81.8%)	38 (88.4%)	0.391	32 (94.1%)	30 (88.2%)	0.388	68 (87.2%)	68 (88.2%)	0.830
T3	8 (18.2%)	5 (11.6%)		2 (5.9%)	4 (11.8%)		10 (12.8%)	9 (11.7%)	
Histologic grade									
Well/moderate	29 (65.9%)	27 (62.8%)	0.761	21 (61.8%)	25 (73.5%)	0.300	34 (43.6%)	43 (55.8%)	0.127
Poor/NS	15 (34.1%)	16 (37.2%)		13 (38.2%)	9 (26.5%)		44 (56.4%)	34 (44.2%)	
Lymph node ratio									
≤1/3	20 (45.5%)	16 (37.2%)	0.067	21 (61.8%)	22 (64.7%)	0.801	35 (44.9%)	44 (57.1%)	0.127
>1/3	24 (54.5%)	27 (62.8%)		13 (39.2%)	12 (35.3%)		43 (55.1%)	33 (42.9%)	
Brain metastasis									
BM	26 (59.1%)	6 (14.0%)	0.000	21 (61.8%)	9 (26.5%)	0.003	47 (60.3%)	15 (19.5%)	0.000
NBM	18 (40.9%)	37 (86.0%)		13 (38.2%)	25 (73.5%)		31 (39.7%)	62 (80.5%)	

BM, brain metastasis; NBM, no brain metastasis; NS, not stated.

**Table 3:** Multivariate cox regression analysis between miR-4270 expression and BM LAD patients.

Variable	Discovery group (n = 87)			Validation group (n = 68)			Full group (n = 155)		
	95%CI	*RR*	*P*	95%CI	*RR*	*P*	95%CI	*RR*	*P*
Sex (male vs. female)	0.487–2.181	1.024	0.917	0.677–3.107	1.451	0.338	0.753–2.158	1.275	0.366
Age (≤60 vs. > 60 years)	0.228–0.992	0.476	0.048	0.420–1.985	0.913	0.818	0.452–1.234	0.747	0.254
Tumor stages (T1+ T2 vs. T3)	0.422–3.478	0.722	0.648	0.366–7.220	1.626	0.523	0.535–2.814	1.227	0.630
Histologic grade (Well/moderate vs. Poor/NS)	0.364–1.686	0.784	0.533	0.320–1.671	0.732	0.459	0.369–1.026	0.615	0.063
Lymph node ratio (≤ 1/3 vs. > 1/3)	1.027–5.201	2.311	0.043	0.441–2.110	0.965	0.928	0.703–2.033	1.195	0.511
miR-4270 expression levels	0.107–0.660	0.265	0.004	0.089–0.490	0.208	0.000	0.133–0.437	0.241	0.000

RR, Relative Risk

**Table 4:** Correlation between miR-423-3p expression and the clinicopathological features of LAD patients with and without BM.

Characteristics	miR-423-3p expression levels of discovery group			miR-423-3p expression levels of validation group			miR-423-3p expression levels of full group		
	Low (n = 44)	High (n = 43)	*P*	Low (n = 34)	High (n = 34)	*P*	Low (n = 78)	High (n = 77)	*P*
Gender									
Male	24 (54.5%)	26 (60.5%)	0.577	20 (58.8%)	22 (64.7%)	0.618	44 (56.4%)	48 (62.%)	0.453
Female	20 (45.5%)	17 (39.5%)		14 (41.2%)	12 (35.3%)		34 (43.6%)	29 (37.7%)	
Age									
≤ 60	20 (45.5%)	27 (62.8%)	0.105	15 (44.1%)	14 (41.2%)	0.806	35 (44.9%)	41 (53.2%)	0.297
> 60	24 (54.5%)	16 (37.2%)		19 (55.9%)	20 (58.8%)		43 (55.1%)	26 (46.8%)	
Tumor stage									
T1+ T2	40 (90.9%)	34 (79.1%)	0.121	32 (94.1%)	30 (88.2%)	0.388	72 (92.3%)	64 (83.1%)	0.081
T3	4 (9.1%)	9 (20.9%)		2 (5.9%)	4 (11.8%)		6 (7.7%)	13 (16.9%)	
Histologic grade									
Well/moderate	27 (62.8%)	29 (65.9%)	0.554	24 (70.6%)	22 (64.7%)	0.604	41 (52.6%)	36 (46.8%)	0.469
Poor/NS	17 (54.8%)	14 (45.2%)		10 (29.4%)	12 (35.3%)		37 (47.4%)	41 (53.2%)	
Lymph node ratio									
≤1/3	21 (58.3%)	15 (41.7%)	0.224	22 (64.7%)	21 (61.8%)	0.801	43 (55.1%)	36 (46.8%)	0.297
> 1/3	23 (45.1%)	28 (54.9%)		12 (35.3%)	13 (39.2%)		35 (44.9%)	41 (53.2%)	
Brain metastasis									
BM	5 (11.4%)	27 (62.8%)	0.000	9 (26.5%)	21 (61.8%)	0.003	14 (17.9%)	28 (62.3%)	0.000
NBM	39(88.6%)	16 (37.2%)		25 (73.5%)	13 (38.2%)		64 (82.1%)	29 (37.7%)	

BM, brain metastasis; NBM, no brain metastasis; NS, not stated.

**Table 5:** Multivariate cox regression analysis between miR-423-3p expression and BM LAD patients.

Variable	Discovery group (n = 87)			Validation group (n = 68)			Full group (n = 155)		
	95%CI	*RR*	*P*	95%CI	*RR*	*P*	95%CI	*RR*	*P*
Sex (male vs. female)	0.474–2.197	1.020	0.959	0.780–3.625	1.681	0.185	0.683–1.994	1.167	0.572
Age (≤60 vs. > 60 years)	0.302–1.333	0.634	0.229	0.345–1.735	0.774	0.534	0.515–1.413	0.853	0.537
Tumor stages (T1+ T2 vs.T3)	0.344–2.896	0.999	0.998	0.225–4.369	0.992	0.991	0.407–2.135	0.932	0.867
Histologic grade (Well/moderate vs. Poor/NS)	0.379–1.828	0.833	0.648	0.408–2.350	0.980	0.963	0.385–1.082	0.646	0.097
Lymph node ratio (≤ 1/3 vs. > 1/3)	1.054–5.338	2.372	0.037	0.433–2.154	0.966	0.932	0.733–2.130	1.250	0.413
miR-423-3p expression levels	2.024–14.418	5.403	0.001	2.439–12.917	5.613	0.000	2.820–9.509	5.179	0.000

RR, Relative Risk

### miR-4270 and miR-423-3p contributed to brain metastasis *in vivo*

We next analyzed the molecular functions of the differentially expressed miRNAs during BM pathogenesis in a lung adenocarcinoma mouse model. Two LAD cell lines, ANIP-973, expressing a relatively high level of miR-4270 (**Fig 2A**), and NCI H1299, expressing a relatively low level of miR-423-3p (**Fig 3A**), were selected for further experiments. A stable miR-4270-knockdown ANIP-973 cell line (**Fig 2B**) and a stable miR-423-3p-overexpression H1299 cell line (**Fig 3B**) were produced for *in vivo* experiments. Subcutaneous injection of ANIP-973 and H1299 cells into BALB/c mice produced transplanted tumors within one week. Tumor volumes were measured weekly, and mice were euthanized after six weeks. Both miR-4270 knockdown and miR-423-3p overexpression increased the growth of LAD tumors *in vivo* (**Fig 2C**; **Fig 3C)**. Immunohistochemistry (IHC) results indicated that both the downregulation of miR-4270 and the upregulation of miR-423-3p upregulated the cell proliferation marker Ki-67. **(Fig 2D**; **Fig 3D**).

**Fig 2:** Tumor growth and metastasis associated with miR-4270 *in vivo*. (A–B) Levels of miR-4270 in five NSCLC cell lines (left panel), stable miR-4270-knockdown A973 cells (Lenti-Inhibitor), and control A973 cells (Lenti-Control) (right panel). (C) Tumor volumes in mice subcutaneously implanted with stable miR-4270-knockdown A973 cells (left panel) and representative images of endpoint tumor burden, as determined by *in vivo* luciferase imaging (right panel). (D) Representative H&E-stained images and Ki-67 IHC-stained images of the miR-4270-knowckdown xenograft. (E) Representative images of tumor burden, as determined by *in vivo* luciferase imaging of the lung, brain, liver, adrenal gland, and bone. Endpoint H&E staining results for mice subjected to the tail vein injection of stable miR-4270-knockdown A973 cells. Data are presented as the means ± SD of three experiments. ** *P* < 0.01 and * *P* < 0.05.

**Fig 3:** Tumor growth and metastasis associated with miR-423-3p *in vivo*. (A–B) Levels of miR-423-3p in five NSCLC cell lines (left panel), stable miR-423-3p-overexpression H1299 cells (Lenti-Mimic), and control H1299 cells (Lenti-Control) (right panel). (C) Tumor volumes in mice subcutaneously implanted with stable miR-423-3p-overexpression H1299 cells (left panel), and representative images of endpoint tumor burden, as determined by *in vivo* luciferase imaging (right panel). (D) Representative H&E-stained images and Ki-67 IHC-stained images of the miR-423-3p-overexpression xenograft. (E) Representative images of tumor burden, as determined by *in vivo* luciferase imaging of the lung, brain, liver, adrenal gland, and bone. Endpoint H&E staining results for mice subjected to the tail vein injection of stable miR-423-3p-overexpression H1299 cells. Data are presented as the means ± SD of three experiments. ** *P* < 0.01 and * *P* < 0.05.

We then injected 10^6^ luciferase-labeled cells into the tail veins of nude mice. Mice were euthanatized after six weeks. Luciferase activity was used to evaluate the tumor burden in all mouse organs. The lung, liver, adrenal gland, and bone metastasis burdens were significantly higher in the mice injected with miR-4270-knockdown cells or with miR-423-3p-overexpression cells, as compared with the control group (**Figs 2E** and **3E**). As expected, the tail-vein injection of either miR-4270-knockdown ANIP-973 cells or miR-423-3p-overexpression H1299 cells significantly increased BM risk (**Figs 2E** and **3E**). These results suggested that miR-4270 and miR-423-3p play important roles in the LAD growth and metastasis *in vivo*, especially with respect to BM progression.

### miR-4270 and miR-423-3p contributed to the malignant LAD phenotype *in vitro*

To further explore the biological functions of miR-4270 and miR-423-3p, we transferred miR-4270 and miR-423-3p mimics into LAD cells. qRT-PCR results indicated that miR-4270 and miR-423-3p expression levels increased significantly in cells transfected with miRNA mimics (**Fig 4A; Fig 4E**). Transfection of H157 and H1299 cells with the miR-4270 mimic for 48, 72, and 96 hours significantly inhibited cell viability (**Fig 4B**). Cell colony formation and migration ability were also suppressed after transfection with a miR-4270 mimic (**Fig 4C and 4D; S2A Fig**). Transfection of H157 and H1299 cells with the miR-423-3p mimic had the opposite effect: overexpression of miR-423-3p not only enhanced the cell viability, but also increased colony formation and cell migration (**Fig 4F–4H; S2B Fig**).

**Fig 4:** Cell proliferation, colony formation, migration, and invasion. (A) Quantification of miR-4270 expression after transfection with the miR-4270 mimic. (B) The cell growth curve measured by MTS after the transfection of the miR-4270 mimic. All the ODs at 490 were normalized to the starred value (at 0 h). (C–D) Representative images and quantitative results for the migration and colony formation assays after the transfection with the miR-4270 mimic. **(E**) Quantification of miR-423-3p expression after the transfection of the miR-423-3p mimic. (F) The cell growth curve, as measured by MTS, after the transfection of the miR-423-3p mimic. All the ODs at 570 were normalized to the starred value (at 0 h). (G–H) Representative images and quantitative results for the migration and colony formation assays after the transfection with the miR-423-3p mimic. Data are presented as the means ± SD of three experiments. ** *P* < 0.01 and * *P* < 0.05.

We transfected LAD cells with miR-4270 and miR-423-3p inhibitors to validate our mimic-transfection results. As expected, the inhibition of miR-4270 expression enhanced the malignant phenotype of LAD *in vitro*, increasing cell growth, colony formation, and cell migration (**Fig 5A–5D; S2C Fig**). In contrast, the inhibition of miR-423-3p expression in LAD cells significantly suppressed the malignant phenotype (**Fig 5E–5H; S2D Fig**). These results indicated that miR-4270 inhibited the proliferation, migration, and invasion of LAD cells *in vitro*, while miR-423-3 promoted these malignant activities.

**Fig 5:** Cell proliferation, colony formation, migration, and invasion. (A) Quantification of miR-4270 expression after transfection with the miR-4270 inhibitor. (B) The cell growth curve, measured by MTS, after the transfection of the miR-4270 inhibitor. All ODs at 570 nm were normalized to the starred value (at 0 h). (C-D) Representative images and quantitative results for the migration and colony formation assays after the transfection of the miR-4270 inhibitor. (E) Quantification of miR-423-3p expression after the transfection of the miR-423-3p inhibitor. (F) The cell growth curve, measured by MTS, after the transfection of the miR-423-3p mimic. All ODs at 570 nm were normalized to the starred value (at 0 h). (G–H) Representative images and quantitative results for the migration and colony formation assays after the transfection of the miR-423-3p inhibitor. Data are presented as the means ± SD of three experiments. ** *P* < 0.01 and * *P* < 0.05.

### Identification of miR-4270 and miR-423-3p targets

To identify proteins regulated by miR-4270 and miR-423-3p, we first searched the publicly available databases TargetScan, PicTar, and miRanda. We found that 3’-UTR of one of the significantly differentially expressed genes, *MMP-19*, included a sequence complementing miR-4270. Similarly, a sequence complementing miR-423-3p appeared in the 3’-UTR of another differentially expressed gene, *P21*. Based on this result, as well as our transcriptome analysis, *MMP-19* and *P21* were selected as potential miRNA targets and further analyzed (**Fig 6A and 6B**).

**Fig 6:** Putative target genes of miR-4270 and miR-423-3p. (A–B) The predicted miR-4270 binding site in the 3’-UTR of *MMP-19* (left panel), and the predicted miR-423-3p binding site in the 3’-UTR of *P21* (right panel). (C–D) Quantification of (C) *MMP-19* mRNA expression and (D) *P21* mRNA expression after the transfection of the miRNA mimic or inhibitor. (E–F) Quantification of (E) *MMP-19* protein expression and (F) *P21* protein expression after the transfection of the miRNA mimic or inhibitor. (G–H) Results of luciferase reporter assay, after (G) the co-transfection of cells with miR-4270 and the pGL3 construct containing *MMP19* with either a WT or a MT 3’-UTR region, or (H) the co-transfection of cells with miR-423-3p and the pGL3 construct containing *P21* with either a WT or a MT 3’-UTR region. Results were normalized to those of cells co-transfected with the negative control mimic (NC) and the pGL3 construct containing either a WT or a MT *MMP19* or *P21*. (I–J) Immunohistochemistry of *MMP-19* and *P21* in the tumor tissues of nude mice treated with (I) the miR-4270-knockdown xenograft or (J) the miR-423-3p-overexpression xenograft. Data are presented as the means ± SD of three experiments. ** *P* < 0.01.

Transfection with miR-4270 and miR-423-3p mimics decreased the mRNA and protein expression levels of *MMP-19* and *P21*, respectively (**Fig 6C and 6D**). Conversely, the mRNA and protein expression levels of *MMP19* and *P21* were significantly increased after transfection with inhibitors of miR-4270 and miR-423-3p, respectively (**Fig 6E and 6F**). We next used a dual-luciferase reporter assay investigate the regulatory effects of miR-4270 on *MMP-19*, and of miR-423-3p on *P21*. The overexpression of miR-4270 in H157 cells suppressed the activity of the luciferase reporter fused to the 3’-UTR of wild-type *MMP19*, but not the activity of the luciferase reporter fused to the 3’-UTR of mutant *MMP19*. Similarly, miR-423-3p suppressed the activity of the luciferase reporter fused to the 3’-UTR of wild-type *P21*, but not the activity of the luciferase reporter fused to the 3’-UTR of mutant *P21* (**Fig 6G and 6H**). Moreover, *MMP-19* was more strongly expressed in upregulated miR-4270 xenograft tumors than in controls expressing miR-4270 normally (**Fig 6I**). In contrast, *P21* was more weakly expressed in miR-423-3p-overexpressed cell-derived tumors than in tumors expressing normal levels of miR-423-3p (**Fig 6J**). Thus, both our *in vitro* and *in vivo* results suggested that *MMP19* was a direct target of miR-4270, and that *P21* was a direct target of miR-423-3p.

Rescue experiments were performed to confirm that *MMP-19* and *P21* were the functional targets of miR-4270 and miR-423-3p, respectively. H157 cells were transfected with a miR-4270 mimic, a control plasmid, or a plasmid expressing *MMP-19*. The downregulation of *MMP-19* and the reduced cell migration caused by miR-4270 overexpression were markedly reversed after transfection with the *MMP-19* plasmid (**Fig 7A and 7B**). To further explore the clinical significance of *MMP-19* expression, we used IHC analysis to evaluate differences in *MMP-19* expression among identical formalin-fixed paraffin-embedded (FFPE) tissue types from the 68 LAD patients. We found that *MMP-19* expression was significantly higher in tissues from BM LAD patients, as compared to NBM LAD patients (**Fig 7C; S5 Table**). Moreover, *MMP-19* expression was positively correlated with histologic grade (**S5 Table**). We also performed a Spearman correlation coefficient analysis to measure the association between miR-4270 expression and *MMP-19* expression in LAD tissues. miR-4270 expression levels were inversely correlated with *MMP-19* expression levels (**Fig 7D**). This was consistent with the observation that *P21* mRNA and endogenous protein expression levels in the H1299 cell line decreased after mimic transfection, and were rescued after transfection with the *P21* expression plasmid (**Fig 7E**). Thus, the migration and invasion induced by mimic transfection were reversed by transfection with the *P21* expression constructs (**Fig 7F**). *P21* staining was negative or weak in NBM LAD tissue, but positive in BM LAD tissue (**Fig 7G; S5 Table**). Furthermore, *P21* expression was negatively correlated with the LAD lymph node metastasis ratio (**S5 Table**). Finally, Spearman analysis indicated that miR-423-3p expression levels were inversely correlated with *P21* levels in the 68 LAD specimens (**Fig 7H**).

**Fig 7:** Rescue assay of miR-4270 and miR-423-3p. (A) The mRNA and protein expression levels of *MMP-19*. (B) The results of the migration assay after the co-transfection of cells with the miR-4270 mimic and the pEGFP-C1 plasmid containing an *MMP-19* CDS sequence. (C) *MMP-19* protein expression, as measured by immunohistochemical staining, in LAD samples. (D) Spearman correlation analysis showing the negative correlation between *MMP-19* and miR-4270 expression. (E) The mRNA and protein expression levels of *P21*. (F) The results of the migration assay after the co-transfection of cells with the miR-423-3p mimic and pEGFP-C1 plasmid containing a *P21* CDS sequence. (G) *P21* protein expression, as measured by immunohistochemical staining, in LAD samples. (H) Spearman correlation analysis showing the negative correlation between *P21* and miR-423-3p expression. Data are presented as the means ± SD of three experiments. ** *P* < 0.01.

## Discussion

BM is becoming increasingly prevalent as systemic diseases become better controlled, because large molecules, such as antibodies, are used to treat primary cancers [26,27]. Due to the blood-brain barrier (BBB) and the unique brain microenvironment, novel approaches are required to treat BMs [18,26]. The ability to identify patients at risk of BM might lead to novel prophylactic interventions, mitigating morbidity and mortality. However, previous efforts to reveal the etiopathogenesis of NSCLC BM, and to predict which NSCLC patients will develop BM [26], have been mostly unsuccessful.

Recently, miRNAs have emerged as a prominent class of gene regulators [1,2]. Bioinformatics analyses have suggested that 30% of all mammalian protein-coding genes may be regulated by miRNAs [3]. Due to the multimodal downstream signaling effect, miRNAs may be useful for human cancer prognoses as well as treatments [4,5]. Indeed, some studies have investigated the mechanistic roles of miRNAs in the BM phenotype [22,23]. Several differentially expressed miRNAs have previously been identified in NSCLC patients (e.g. miR-1, miR-137, and Let-7a) [28–29]. However, few studies have examined the association between miRNA expression and BM risk in NSCLC patients.

Although some BM-associated miRNAs (e.g. miR-328 and miR-326) in NSCLC patients using miRNA arrays [22,30], sample sizes in these previous studies were relatively small (n = 12). Here, we used miRNA array profiling and real-time PCR validation to identify miRNAs associated with BM in a relatively large sample (n = 155). Notably, most of the differentially expressed miRNAs identified in this study differed from those previously reported [22]. Of these miRNAs, five (miR-193a-5p, miR-210, miR-214, miR-423-3p, and miR-423-5p) were significantly upregulated in BM LAD as compared to NBM LAD, and one miRNA (miR-4270) was significantly downregulated. In addition, the mature products of miR-4270 and miR-423-3p were significantly differentially expressed in the BM LAD tissues as compared to the NBM LAD tissues. miR-4270 expression levels in BM LAD patients were significantly lower than in NBM LAD. However, higher levels of miR-423-3p expression were significantly correlated with increased brain metastases. Multivariate cox proportional hazard regression analysis of each of these parameters indicated that low miR-4270 expression and high miR-423-3p expression were significantly unfavorable prognostic factors for LAD, independent of BM. Therefore, the downregulation of miR-4270 and the upregulation of miR-423-3p in BM-positive patients suggested that these miRNAs might be involved in ‘‘brain-seeking” metastatic potential [31,32]. That is, miR-4270 and miR-423-3p may be associated with the pathogenesis of BM from primary LAD, and are thus potential biomarkers.

Here, miR-4270 downregulation and miR-423-3p upregulation were associated with the development of BM from primary LAD. Intriguingly, previous studies have shown that miR-4270 is upregulated in breast cancer and the peritoneal metastasis of gastric cancer [33,34], indicating that different levels of miR-4270 expression might be associated with different cancers. In addition, miR-423-3p downregulation has been reported during NSCLC lymph node metastasis [35], suggesting that different levels of miR-423-3p expression might be associated with different stages of NSCLC metastasis. miR-423-3p might be a useful biomarker of the difference between hereditary and non-hereditary breast cancers [36]. miR-423-3p might also contribute to LAD tumor progression through similar signaling pathways to those as observed in laryngeal hepatocellular carcinomas [37,38].

The role of miRNAs in the biology of BMs has been established in previous studies of various primary tumor types [39–42]. In lung cancer, MiRNA-378 promotes brain metastases in NSCLC by upregulating *MMP-7*, *MMP-9*, and *VEGF* and downregulating *Sufu*; these genes are critically involved in angiogenesis and extracellular matrix invasion [43]. miRNA-145 downregulation leads to LAD progression, and promotes BM formation [44]. Similarly, changes in miR-1258 expression are directly correlated with the upregulation of heparanase, a prometastatic enzyme found in BM breast cancer cells known to degrade heparan sulfate chains; this degradation affects the cytoskeleton and renders cells more capable of crossing the BBB [45]. Our clinical analyses and mouse models both suggested that miR-4270 and miR-423-3p not only play an important role in BM pathogenesis, but are potential RNA markers of NSCLC patients at a high risk for BM. The miRNAs identified herein are potential diagnostic markers and targets for BM NSCLC drug therapy.

Our cell viability, migration, and colony formation assays indicated that both the downregulation of miR-4270 and the upregulation of miR-423-3p increased cell proliferation and migration. The molecular functions of the putative target genes of miR-4270 and miR-423-3p (*MMP19* and *P21*, respectively) have been well characterized [46−52]. Here, the correlations between miRNA and gene expression in the LAD patients supported the modulation of *MMP-19* and *P21* by miR-4270 and miR-423-3p, respectively. *MMP-19* and *P21* expression levels differed between BM LAD patients and NBM LAD patients.

To our knowledge, this is the first study to demonstrate that *MMP19* and *P21* are involved in the BM pathogenesis in LAD patients. However, with the exception of p21 and MMP19, little in known about the proteins associated with the signaling mechanisms that mediate BM. In future work, we therefore aim to investigate the relationship between other signaling pathways and brain metastasis.

In summary, our miRNA array screening identified several miRNAs associated with BM in LAD. Downregulation of miR-4270 or upregulation of miR-423-3p significantly increased cell proliferation, colony formation, and cell migration *in vitro*. miR-4270 and miR-423-3p increased the risk of BM in mouse models by targeting *MMP19* and *P21*, respectively. Our results suggested that miR-4270 and miR-423-3p are potential diagnostic markers and drug targets, which may improve predictions of BM risk as well as the clinical treatment of LAD patients.

## Materials and methods

### Clinical tissue samples

We enrolled 155 LAD patients in this study. In all cases, LAD was histologically-confirmed between 2003 and 2008 at the Cancer Hospital, Chinese Academy of Medical Sciences (Beijing, China). Of these patients, 62 developed BM. The remaining 93 were classified as NBM. All patients underwent surgical resection followed by adjuvant therapy, according to the standard of care. Formalin-fixed paraffin-embedded (FFPE) specimens were collected from each patient. Two pathologists independently evaluated the histologic tumor type, tumor grade, and tumor percentage using hematoxylin and eosin (H&E)-stained specimens. The clinical characteristics of the patients are summarized in Table 1. Written informed consent was obtained from each patient for the use of their biological materials. This study was approved by the Institutional Review Board of the Cancer Hospital of the Chinese Academy of Medical Sciences.

### Cell culture and transfection

Human LAD cell lines A549, NCI-H1299, NCI-H157, ANIP-973, and GLC-82 were obtained from the Cell Culture Center of Peking Union Medical College (Beijing, China) and the Typical Culture Cell Bank of the Chinese Academy of Sciences (Shanghai, China). DNA typing of the H157 cells indicated that this cell line was an exact match to the cell line in the cell bank. The NCI-H157 cells corresponded to the CRL-5802 cells in the DSMZ database; multiple alleles were not detected in this cell line. The STRs in the H157 cells were compared with the STRs in all cell lines from the ATCC, DSMZ, JCRB, and RIKEN databases. However, the H157 cells could not be matched with any cell line in any databank. Human embryonic kidney (HEK) 293T cells were purchased from the ATCC (Manassas, VA). Human LAD cell lines were cultured in RPMI-1640 medium, and HEK 293T cells were cultured in DMEM supplemented with 10% fetal bovine serum (FBS; Gibco-BRL, Grand Island, NY). Both sets of cells were maintained in a humidified atmosphere with 5% CO_2_ at 37°C. All endogenous mature miRNA mimics and inhibitors were purchased from RiboBio (Guangzhou, China). miRNA mimics, control RNAs, inhibitors, control inhibitors, and plasmids were transfected using Lipofectamine 2000 (Invitrogen), following the manufacturer’s protocols.

### RNA extraction, qRT-PCR, and plasmid construction

Total RNA was extracted from cells and tissues using TRIzol reagent (Invitrogen). First-strand cDNA was synthesized by using MMLV reverse transcriptase (Promega), following the manufacturer’s instructions. PCRs were performed using *Taq* polymerase (Takara) with the specific primers for *MMP-19* (forward: 5’-CTTCAGCAGCTACCCCAAAC-3’; reverse: 5’- CCGTACCTGAGGGAGTGGTA-3’; *P21* (forward: 5’- TTAGCAGCGGAACAAGGAGT-3’; reverse: 5’-GCCGAGAGAAAACAGTCCAG-3’;), and *GAPDH* (as the internal control; forward: 5’-TCTCTG CTCCTCCTGTTC-3’; reverse: 5’-GGTTGAGCACAGGGTACTTTATTGA-3’;). miRNAs were detected using stem-loop primers purchased from Ribobio (Guangzhou, China), following the manufacturer’s instructions. *GAPDH* and *U6* small nucleolar RNAs were used for normalization. qRT-PCRs were performed with the QuantiTect SYBR Green PCR Kit (Takara) on a StepOne Real-Time PCR System (Applied Biosystems). Relative expression levels were calculated by using the 2^−ΔΔCt^ method in Biorad CFX Manager v3.1. The plasmids pDonR223-MMP-19 and pDonR223-P21, carrying human *MMP-19* and *P21*, respectively, were purchased from Axybio Bio-Tech Co., Ltd. (Changsha, China). The complete coding sequence of human *MMP-19* (EMBL accession no. BC050368;) and *P21* (EMBL accession no. BC001935) were amplified from the pDonR223-MMP-19 and pDonR223-P21 plasmids, respectively. The PCR products of *MMP-19* and *P21* were digested separately with the pEGFP-N1 plasmid using *Xho I* and *Hind III*. Fragments were purified and ligated with T4 DNA ligase. The ligated products were transformed into TOP10 competent cells, and positive clones were named either pEGFP-N1-MMP-19 or pEGFP-N1-P21.

### MicroRNA microarray assay and target prediction

Total RNAs were analyzed with μParaflo MicroRNA microarray assays (LC Sciences). The array probes were designed based on miRBase v10.0 (www.mirbase.org). All procedures were performed as stipulated on the LC Sciences website (www.lc-bio.com). RNA samples were also sent to CapitalBio Corp. miRNA microarray experiments were performed using GeneChip miRNA 1.0. All procedures were performed as stipulated on the CapitalBio website (www.capitalbio.com). Sequences were clustered using Cluster 3.0, and visualized with TreeView. Bioinformatics analysis was performed with PicTar (pictar.mdc-berlin.de]), miRanda (www.microrna.org), and TargetScan (www.targetscan.org). Fold change and *P*-value were calculated for each miRNA.

### Luciferase miRNA target reporter assay

For the *MMP-19* and *P21* 3′-UTR luciferase assays, we constructed dual-luciferase vectors (pmiR-RB-REPORT dual-luciferase vector) containing either wild-type or mutant miR-4270 or miR-423-3p binding sites in the 3′-UTRs of *MMP-19* or *P21*, respectively. Mutant binding sites were constructed by substituting four nucleotides in the seed region. NCI-H157 cells were co-transfected with the luciferase reporter gene constructs and miR-4270, and NCI-H1299 cells were co-transfected with the luciferase reporter gene constructs and miR-423-3p. Both cells lines were also co-transected with the luciferase reporter gene constructs and negative control oligonucleotides (miR-NC). After 48 h, cells were lysed and luciferase activity was measured using the Dual-Luciferase Reporter Assay System (Promega). A plasmid containing an expression cassette for Renilla luciferase, pRenilla, was co-transfected and used to normalize the firefly luciferase values expressed by the luciferase reporter gene constructs.

### Cell proliferation assay

Cell proliferation was evaluated using 3-(4,5-dimethylthiazol-2-yl)-5- (3-carboxymethoxyphenyl)-2-(4-sulfophenyl)-2H-tetazolium, following the manufacturer’s instructions. Briefly, an optimal density (5 × 10^3^ cells/mL) of cells in 200 μL of culture medium was added to each well in 96-well culture plates. After 0–96 h of culture, 20 μL of MTS solution was added to each well, and plates were incubated at 37°C for 2 h. The optical density of each sample was immediately measured at 570 nm using a microplate reader (BioRad).

### Colony formation assay

We seeded 1×10^3^ cells were seeded into 100-mm culture plates, and incubated the plates at 37°C under 5% CO_2_ for 2 weeks. Plates were cultured in duplicate. The colonies which total numbers of individuals are more than 50 were counted. After washing with pre-cooled PBS, cultures were fixed with pre-cooled methanol for 20 min, and then stained with crystal violet for 15 min.

### Cell invasion and migration assays

The invasion assay was performed using 24-well Millicell hanging cell culture inserts, consisting of an 8-μm PET membrane (Millipore) coated with BD Matrigel Basement Membrane Matrix. The invasion assay was performed following. Briefly, cells were trypsinized and resuspended in 1640 medium without FBS. The, 5 × 10^4^ cells were added to the upper chamber of each well, while 500 μL of 1640 medium containing 20% FBS was added to the lower chamber. After incubation for 12 h at 37°C, cells on the upper membrane surface were removed by careful wiping with a cotton swab, and the filters were fixed by treatment with methanol for 20 min. Filters were then stained with a 0.1% crystal violet solution for 20 min. Invasive cells adhering to the undersurface of the filter were counted (using five high-power fields) with an inverted microscope. The migration assay was identical to the invasion assay, except that no Matrigel was used.

### Western blotting analysis

Cells were harvested and protein extracts were obtained by lysing the cells with lysis buffer [1% NP-40, 250 mm NaCl, 50 mM Tris-HCl, 10 mM EDTA, and 1 mM DTT, supplemented with a complete protease inhibitor tablet (Sigma, Inc)]. Equal amounts of protein were electrophoresed on 10% SDS–PAGE gels and then transferred to PVDF membranes. After blocking with 5% bovine serum albumin (BSA), membranes were probed with anti-MMP-19, anti-P21 (Abcam), and anti-β-actin (Santa Cruz Biotechnology, Inc.), followed by incubation with a horseradish peroxidase-conjugated secondary antibody [goat-anti-mouse IgG (1:2,000) and goat-anti-rabbit IgG (1:3,000)]. Proteins were visualized with Image Reader LAS 4000 (Fujifilm) and analyzed with Multi Gauge v3.2.

### Generation of stable cell lines

Recombinant lentiviral vectors expressing low levels of miRNA-4270 (miRNA-4270-knockdown), high levels of miRNA-423-3p (miRNA-423-3p-overexpression), or an irrelevant sequence were purchased from Hanbio Biotechnology (Shanghai, China). In addition to the lentiviral expression vectors, we used luciferase and puromycin reporter genes, driven by the EF1α promoter, to indicate infection efficiency. To construct lentiviral vectors, the precursor sequence for miRNA-4270 (pre-mir4270), sponge miRNA-423-3p, and the irrelevant sequence (negative control) were inserted into pHBLV-U6-MCS-EF1α-Luc-T2A-puromycin lentiviral vectors. The recombinant lentiviruses were packaged via the co-transfection of HEK-293T cells with pSPAX2 and pMD2.G using LipoFiter reagent. Supernatants with lentiviral particles were harvested 48 and 72 h after transfection and filtered through 0.45-μm cellulose acetate filters (Millipore, USA). Recombinant lentiviruses were concentrated with ultracentrifugation. To establish stable cell lines, ANIP-973 and NCI-H1299 cells were transducted with lentiviruses (MOI of ~5) in the presence of 5 μg/mL polybrene. Each supernatant was removed after 24 h and replaced with fresh complete culture medium. Infection efficiency was validated with qRT-PCR 96 h after infection. Cells were incubated with 2 μg/mL puromycin for 2 weeks.

### Tumorigenicity and metastasis assay *in vivo* using bioluminescence imaging

All animals used in these experiments were treated humanely, in compliance with the “Guide for the Care and Use of Laboratory Animals”, the Institute of Laboratory Animal Resources, National Institutes of Health, and according to the Animal Experiment Guidelines of Samsung Biomedical Research Institute. The effects of miR-4270 and miR-423-3p on the tumorigenic and metastatic potentials of LAD cells were analyzed in orthotopic and systemic metastasis *in vivo* models. To construct the orthotopic model, 4–6-week-old BALB/c nude mice were subcutaneously injected in the right hip with 1×10^6^ transfected cells. To construct the experimental metastasis *in vivo* model, transfected cancer cells (1×10^6^ cells in 100 μL of HBSS) were directly injected into the tail vein. Six weeks later, the tumor colonies in the subcutaneous tissues were observed using H&E staining and histological examination. Bioluminescence images were collected to assess the growth and metastasis of the implanted tumor cells. To quantify the *in vivo* bioluminescence signals, mice were anesthetized with isoflurane before *in vivo* imaging, and D-luciferin solution (*in vivo* imaging solutions, PerkinElmer; 150 mg/kg in PBS) was intravenously injected into both the orthotopic and systemic xenograft mouse models. Bioluminescence images were acquired with the IVIS Spectrum imaging system (PerkinElmer) 2–5 min after injection. Captured images were quantified using the Living Image software package (Perkin Elmer/Caliper Life Sciences), by measuring the photon flux (photons/s/cm^2^/steradian) within a region of interest (ROI) drawn around the bioluminescence signal.

### Evaluation of immunohistochemical staining

Immunohistochemical staining was performed on 4 μm-thick slices following the two-step EnVision procedure described for the Dako REAL EnVision Detection System. Slides were incubated with one of three primary antibodies: Ki-67 (1:50, Santa Cruz), MMP-19 (1:50, Abcam) and P21 (1:50, Abcam). After incubation, sliders were re-incubated with the HRP-labeled secondary antibody, and then visualized with diaminobenzidine. The expression levels of MMP-19 in the cytoplasm and P21 in the cytoplasm or nucleus were calculated as the average percentage of positive cells times the intensity of the positive cells under five randomly selected high-power fields. Scores were assigned to the obtained percentages as follows: <5% (0), 5–25% (1), 25–50% (2), 50–75% (3), and >75% (4). For intensity, scores were assigned as follows: no staining (0), light brown (1), brown (2), and dark brown (3). For MMP-19 and P21, scores of 0 and ≥1 were defined as negative and positive, respectively.

### Statistical analysis

All measurement data were expressed as the means ± SD, and all error bars represent the standard deviation of the mean. Student’s *t* tests, *χ*^*2*^ tests, and repeated measures ANOVAs were used to determine statistical significance. The cumulative incidence of BM was estimated with the Kaplan-Meier method, and the differences between the two groups were analyzed with the logrank test. Cox regressions (proportional hazards model) were used for multivariate analysis of prognostic factors. Receiver operating characteristic (ROC) curves and the area under the ROC curve were used to assess the accuracy of the miRNA-based BM predictions. All statistical tests were two-sided. *P* < 0.05 was considered statistically significant. Statistical analyses were performed with SPSS v16.0 (SPSS Inc. USA).

## Supporting information

S1 Fig (A) Kaplan-Meier analysis of BM-free survival based on the expression levels of miR-4270, miR-214, miR-423P-5p, miR-210, miR-193-5p, and miR-423-3p in the 87 patients in the discovery group. (B) Kaplan-Meier analysis of BM-free survival based on the expression levels of miR-4270, miR-214, miR-423-5p, miR-210, miR-193-5p, and miR-423-3p in the 68 patients in the validation group.
(TIF)

S2 Fig (A–B) The results of the migration assay after cells were transfected with (A) the miR-4270 mimic or (B) the miR-423-3p mimic. (C–D) The results of the migration assay after cells were transfected with (C) the miR-4270-knockdown GLC82 cells or (D) the miR-423-3p-knockdown A973 cells. ** *P* < 0.01 and * *P* < 0.05.
(TIF)

S1 Table Univariate cox regression analysis of BM LAD patients. (DOCX)

S2 Table Multivariable logistic regression model, predicting BM in LAD patients (in the discovery group) based on miRNAs. (DOCX)

S3 Table Multivariable logistic regression model, predicting BM in LAD patients (in the validation group) based on miRNAs. (DOCX)

S4 Table Multivariable logistic regression model, predicting BM in LAD patients (in the discovery and validation groups combined) based on miRNAs. (DOCX)

S5 Table Correlation between *MMP-19* and *P21* protein expression and the clinicopathological features of LAD patients with and without BM. (DOCX)

S1 Data Differences in miRNA expression profiles between the 32 BM LAD patients and the 55 NBM LAD patients. (XLS)
